The article "The Influence Mechanism of Education on Health from the Sustainable Development Perspective" was published in 2022. Journal: J Environ Public Health.

# The Influence Mechanism of Education on Health from the Sustainable Development Perspective

**DOI:** 10.1155/2022/7134981

**Published:** 2022-07-20

**Authors:** Hui Hui

**Affiliations:** Capital University of Economics and Business, Beijing, China

## Abstract

Good health and quality education are two important goals of the Sustainable Development Goals (SDGs). More and more people pay attention to physical and mental health in a pandemic age. Previous studies have paid more attention to the relationship between socioeconomic status and health, and also scholars at home and abroad have not reached a consistent conclusion on how education affects health. In this study, we try to explore the relationship between education and health from the sustainable development perspective and its internal influence mechanism through the data of China General Social Survey (CGSS) in 2015 and 2017, according to Grossman's health demand model. The results indicated that from the junior high school education, physical health improved with the increase of the education level, but this effect was gradually weakened. The relationship between education and mental health is not a simple linear relationship but an inverted U-shaped change. After 16 years of education, mental health gradually decreases. Compared with women and rural population, men and urban population have better health. Education leads to labor market segmentation, which makes people with different education levels in different social structure positions, resulting in differentiation of lifestyles, psychology, and social interaction, and this ultimately leads to health inequality. Education indirectly improves people's health by changing healthy behaviors, cultivating healthy psychology, and strengthening social interactions.

## 1. Introduction

Since the 21st century, the study of health inequality has been highly concerned by the global community. The World Health Organization (WHO), the World Bank (WB), the United Nations Development Programme (UNDP), and many governments have actively invested in human, material, and financial resources to study health inequality through economic, social, and psychological dimensions in a diverse global background. The influencing factors of health inequality have always been an important part of academic research, mainly including two aspects: social demographic characteristics and socioeconomic status, especially the latter. The health of groups with higher socioeconomic status is usually better than that of groups with lower socioeconomic status [1, 2]. The commonly used socioeconomic status indicators are income, occupation, and education. Education has a more fundamental role than income and occupation [3–7].

Studies suggest that people with higher education live longer, having a healthier physical and psychological condition, which is called “education gradient in health” emphasized by economics, sociology, psychology, and epidemiology. Previous studies mostly focused on the people of developed countries, and the research conclusions may not be fully applicable to developing countries. Based on this consideration, what is the relationship between education and health in China? If education has a significant impact on health, what is the mechanism behind? Therefore, this study attempts to answer whether education has an impact on people's health through Chinese experience, so as to clarify the influence mechanism of education on health inequality and provide further reference for the government to formulate education and health policies.

## 2. Literature Review

From the Alma-Ata Declaration of 1978, the United Nations (UN) called on all countries in the world to work together to achieve the goal of “Health for All in 2000.” It defines the importance of main health care and delineating governments duties for health. Since then, people's understanding of health has been expanding. The relationship between education and health has been one of the most important topics in western academia, and a large number of empirical research results have been formed.

Winkleby et al. [8] found that education has a close relationship with people's cholesterol content. The people who have higher education got a lower risk of excessive cholesterol. Pappas [9] found that the mortality rate of white males with higher education was significantly lower than the white males without higher education in the same period in the United States in 1960–1986. Ross and Wu [10] found that people with higher education know how to use the healthcare services better, and their self-rated health is better. Ross and Mirowsky [5] found that highly educated people feel more substantial and valuable at work, and their ability to regulate life and health is significantly stronger, which explains why education is the most important factor affecting people's health.

Compared with a large number of literature studies on the relationship between education and physical health, the academic circle has relatively little discussion on the relationship between education and mental health. A small number of studies show that the relationship between education and mental health is also complicated, and there are two completely different views. First, education has a significant positive impact on mental health. Rates of schizophrenia and depression have fallen significantly among highly educated people, both in developed western countries and in less developed regions, such as Latin America. The positive emotions and self-measured mental health factor score of illiterate and primary school education residents were significantly lower than those of high school education or above. Educational achievement can protect individual mental health and reduce mental health risk effectively. Second, education has a significant negative impact on mental health. People with a higher education level have higher self-expectations. Once they encounter difficulties or crises such as unemployment, income, and decline in professional status, it is difficult to realize their self-expectations. They may have a greater sense of pressure and loss, forming negative emotions such as tension, anxiety, and pessimism, leading to a decline in mental health.

In summary, the relationship between education and health at home and abroad has not formed a consistent conclusion yet. The research can be further expanded in China: in the aspect of research object, the previous studies mainly concentrated on the migrant workers, the elderly, and other specific groups, which is lack of a comprehensive discussion of the entire adult group; in terms of content, the previous research focused on the comparative study of groups or regions, and there are few of them on the internal mechanism of education and health in peoples' behaviors and psychology way. Therefore, this study attempts to comprehensively explore the influence mechanism of education on health from the above two aspects by using the data of China General Social Survey (CGSS).

## 3. Theory and Hypothesis

In a very broad sense, there are three possible reasons for the link between health and education. One reason is that poor health leads to low levels of education. Another possibility is that increasing education improves health. Lastly, there may be third factors that increase both education and health. It is important for policy to understand how much of the observed correlation between education and health can be explained by each of these explanations. Subsidies for schooling would only be effective in improving the health of the population if, in fact, education causes health.

There are two representative theories in the study of health inequality: one is “resource substitution theory,” and the other is “reinforcement of advantage theory” [5]. Resource substitution theory believes that as a social resource, education will promote health more significantly in vulnerable groups. Because this group has disadvantages in social resources, it will be more dependent on rare educational resources, thus benefiting more from educational achievements. Resource substitution theory forecasts people's age, injury levels, and a rise in the poorly educated. According to this theory, the educational impact on health is superior for those whose parents are also educated or that the personal education impact on health is unaffected by parental education. And by this theory, education enhances women's well-being more than men's since women's socioeconomic disadvantage forces them to rely more on education to obtain happiness. This theory would help to understand that personal control, healthy lifestyle, job, and economic situations all facilitate the conditional effect of education on health, and these mediators follow the same conditional pattern as education.

On the contrary, reinforcement of advantage theory argues that the promotion of education to health will cause “Matthew Effect” [5, 11], which means individuals with more social resources will benefit more from educational achievements. The method of influencing behavior through regulating the behavior consequences is known as the reinforcement theory. In this theory, a grouping of rewards would reinforce preferred behavior or eliminate undesirable behavior. Selective perception, selective retention, and selective exposure are the three fundamental mechanisms that reinforce this theory. Reinforcement theorists believe that behavior is influenced by the environment, and instead of interior thoughts, the behaviors are measured by reinforces.

These two theories are supported by empirical data in most western countries. Therefore, based on theoretical analysis, we believe that education has a significant positive impact on individual health. Accordingly, we propose hypothesis 1: people with higher levels of education are healthier.

Education is an important human capital and affects access to economic, psychological, and social resources, which in turn affect people's physical and mental health. First, education affects the promotion of socioeconomic status and the accumulation of material returns. Good education improves individual human capital, which can make people occupy a greater advantage in the labor market competition. There is a greater chance of securing a stable, better-paying job in a better environment, and the material rewards of education contribute to maintaining better physical health. Stable work and good income bring people greater psychological satisfaction and happiness and promote the improvement of their mental health level [12]. Secondly, education enables people to acquire more health knowledge and shape a healthy lifestyle. Education also enhances life planning and controls ability, cultivating optimistic life attitude and constructing positive psychological capital. Educated people are more likely to be physically active regularly, drink moderately, avoid obesity, smoke less, and feel more in control of their lives. These good living habits, scientific lifestyle, and positive life attitude can significantly improve physical and mental health [13]. Finally, educational achievement may influence physical and mental health through social support resources. The higher the level of education, the more medical support they receive, such as regular health check-ups. When health problems arise, better medical support services are available to maintain good health. Generally speaking, well-educated people have strong social communication ability, which is conducive to expanding and maintaining social relations with others [14]. In addition, people can obtain more psychological and emotional support from social networks, strengthening their happy experience and maintaining good mental health status [15]. Based on the above analysis, hypothesis 2 is established: education indirectly affects people's physical and mental health through income, lifestyle, and social interaction.

## 4. Materials and Methods

### 4.1. Model Construction

In order to analyze the correlation between education and health, we use Grossman's [16] health demand model to estimate the following regression:

(1) $$\begin{array}{c} H_{i}=C+\alpha E_{i}+\beta X_{i}+\varepsilon , \end{array}$$

where *H*_*i*_ is a measure of individual *i*'s physical and mental health, *E*_*i*_ stands for individual *i*'s years of completed education, *X*_*i*_ is a vector of individual characteristics that includes gender, age, and registration place, *c* is a constant term, and *ε* is the error term. The coefficient on education *α* (also referred to as the education gradient) is the object of interest, and it measures the effect of one more year of education on the particular measure of health.

In order to further clarify the relationship between education and health, as well as the influencing factors, based on the baseline model, three possible influencing factors proposed by existing theories are introduced: income, lifestyle, and social interaction. We estimate the regression as follows:

(2) $$\begin{array}{c} H_{i}=\beta_{0}+\beta_{1}E_{i}+\beta_{2}X_{i}+\beta_{3}Y_{i}+\beta_{4}E_{i}\times I_{i}+\beta_{5}E_{i}\times L_{i}+\beta_{6}E_{i}\times S_{i}+\varepsilon , \end{array}$$

where *H*_*i*_ is a measure of individual *i*'s physical and mental health, *E*_*i*_ stands for individual *i*'s years of completed education, *X*_*i*_ is a vector of individual characteristics, *Y*_*i*_ stands for the influencing factors, such as income, lifestyle, and social interaction. *E*_*i*_ × *I*_*i*_ is the interaction with education and income; *E*_*i*_ × *L*_*i*_ is the interaction with education and lifestyle; *E*_*i*_ × *S*_*i*_ is the interaction with education and social interaction. *β*_0_ is a constant term, and *ε* is the error term.

### 4.2. Data and Measurement

The data we used are from the 2015 and 2017 Chinese General Social Survey (CGSS), which is the first large-scale national, comprehensive, and continuous social survey project in China. The survey covers most provinces and regions in the mainland of China by using the multilevel stratified sampling method. In the survey, since respondents who answered health-related questions were randomly selected, the missing values in this part can be approximately regarded as completely random missing, which can be directly eliminated without further processing. Therefore, the final sample size is 11078.

In the studies of health inequality, the measurements of health include self-rated health, mortality, medical health, and functional health indicators [3]. The dependent variable of this study is physical and mental health. We measure the level of physical health through self-assessment of health. The respondents answered the self-rated health question, “How is your current physical condition?” (1= very unhealthy; 2= relatively unhealthy; 3= general; 4= relatively healthy; 5= very healthy). We treat self-rated health as a binary variable. “very healthy, relatively healthy and fair” is coded as “good health =1.” “Very unhealthy and relatively unhealthy” is coded as “Poor health =0.” We measure the level of mental health through Hopkins Symptoms Check List (simplified version), which consists of 8 questions. Respondents answered from “no, occasionally, sometimes, and often” and assigned a score of 4 to 1. The principal component method was used for factor analysis of the score, and the formula was used to convert the mental health factor value into 1–100 points. The higher the score, the better the mental health.

The independent variable is the level of education. In order to reflect the nonlinear relationship between education levels [17], the five-classification method is used to divide the level of education into 1= without any education; 2= primary school; 3= junior high school; 4= high school; 5= college and above [18]. The control variable is gender (1= male; 0= female), age, and registration place (1= urban; 0= rural).

In this study, the socioeconomic status was measured by personal annual income (logarithmic conversion). Lifestyle was measured by the frequency of physical exercise (1= daily; 2= several times a week; 3= several times a month; 4= several or less a year; 5= never). Social interaction is measured by the frequency of participation in group activities (1= once a week or more; 2= 1 to 3 times a month; 3= attended several times last year; 4= participated once last year; 5= never participated). In order to avoid the sample selection bias caused by population mobility and the estimation error caused by the sample size difference, we add interactions in the model in turn, rather than directly comparing the coefficients of the subsample model [19]. The descriptive statistical results of the data are shown in Table 1.

According to Table 1, in the physical health part, residents' self-rated health level is high. In terms of mental health, the average score of residents' mental health was 90.6. As can be seen, the general mental health of the population is relatively good.

## 5. Empirical Analysis and Results

### 5.1. Analysis of the Influence Mechanism of Education on Physical Health

We use the multiple linear regression method to establish the baseline model first, and then put variables into the baseline model in turn: personal income (personal annual income), lifestyle (physical exercise), social interaction (group activities), and their interactions with education. Then, we test the hypotheses 1–2, respectively, and analyze the influencing factors of education on health. The results are shown in Table 2.

Model 1 shows that education has no significant effect on health in primary education. From the junior high school, education has a significant positive effect on health. Compared with primary school people, junior high school, high school, college, and above people reported good health that was increased by 12.98%, 16.53%, and 17.47%. This shows that education and health are linear, rather than the “inverted U” type. That is, from the junior high school, the health becomes better with the improvement of the education level, but the influence of education on health gradually weakens.

In model 2, the regression coefficient of the years of completed education was 0.127, and it was significant at 0.01 level. That means for every additional year of education, health improves by 13.5%. The empirical results are similar to those of foreign studies [10, 19], and they also confirm the theory of learned effectiveness [20] that education is an ability to acquire effectiveness. Comprehensive model 1 and model 2 show that hypothesis 1 is supported.

Control variables also have an important impact on individual health. In terms of gender, the health advantage of men is obvious, and the health status of men is better than that of women by 13.7%, which is consistent with previous studies [21]. In terms of age, there is a significant negative correlation with physical health; that is, with the increase of age, physical health gradually decreased. In terms of urban-rural differences, there are obvious health differences between urban and rural populations. The advantages of urban population in reporting good health are 1.3 times of rural population, indicating that urban residents are better than rural residents in medical services, health environment, and economic development. These factors significantly improve the health level of urban residents, consistent with previous studies [1].

In model 3, the main effect of personal income has a significant positive impact on health after adding the interaction between education and income. The data showed that for each additional unit of the natural logarithm of personal annual income, the health improved by 18%. In model 4, people who often participate in physical exercise have a healthier physical condition. The data show that the frequency of participating in physical exercise increases by one unit, and the health improved by 1.16 times. In model 5, people with frequent social interaction have a healthier physical condition. The data show that under the interaction of education and group activities, the frequency of participating in group activities increases by one unit, and the health improved by 1.12 times.

Comprehensive models 3, 4, and 5, the years of completed education, have a significant role in promoting self-rated health. However, the main effect coefficient of education is reduced to varying degrees after the interactions of education and income, education and physical exercise, and education and group activities are included. This shows that education affects personal health by affecting the personal income level, lifestyle, and social interaction. Therefore, hypothesis 2 was supported.

### 5.2. Analysis of the Influence Mechanism of Education on Mental Health

Education has a significant effect on mental health (Table 3). After controlling for other variables, Model 1 indicates that the higher the educational level, the better the mental health status. The results of Model 2 show that the relationship between education and mental health is not a simple linear one but an inverted U-shaped curve. With the increase of years of education, the mental health of postgraduates increases first and then decreases. When the years of education reach about 16 years, the mental health of postgraduates gradually decreases. Because the self-expectation level of postgraduates is higher, they are more engaged in administrative management and professional/technical work. They are facing greater work pressure and are easy to form tension and anxiety which will lead to worse mental health. Combined results show that hypothesis 1 is not supported.

Comprehensive model 3, the results showed that income, physical exercise, and community participation all had significant positive effects on mental health. It also suggests that income, physical exercise, and community participation explain part of the difference in the impact of education on mental health, and these three are important mediating factors of education on mental health. Therefore, hypothesis 2 was supported.

## 6. Discussion and Conclusions

Previous studies have paid more attention to the relationship between socioeconomic status and health, and scholars at home and abroad have not reached a consistent conclusion on how education affects physical and mental health. This study uses the data of China's General Social Survey (CGSS) to explore the relationship between education and health, and its internal influence mechanism from the sustainable development perspective. The results indicate that education has a significant promoting effect on physical and mental health whether it is measured by education levels or years of completed education. The study found that from the junior high school education, individual's physical health improved with the increase of the education level, but the growth rate gradually slowed down. The relationship between education and mental health is not a simple linear relationship but an inverted U-shaped change. After 16 years of education, mental health gradually decreases. Compared with women and rural population, men and urban population have better health. This result confirms “reinforcement of advantage theory.” In the impact mechanism, the analysis confirms that education indirectly improves people's physical and mental health by raising income, changing lifestyle, and strengthening social interaction.

The above results suggest that education not only affects individual material returns but also brings nonmaterial returns. Educational achievement is an important factor affecting health, which means that educational inequality leads to health inequality. The trend of health inequality in western countries also exists in China. This study suggests that education leads to labor market segmentation, which makes people with different education levels in different social structure positions, resulting in differentiation of economic status, lifestyle, and social interaction, and this ultimately leads to health inequality.

For those with lower education level, they are difficult to enter the primary labor market who stay more in the secondary labor market or the agricultural sector, engaging in simple and repetitive productive work. There are more unhealthy factors in their working environment, and they have lower return on work and are limited in health care, healthy lifestyle, and social interaction. This means that the low material return brought by education has a negative impact on health. The people with lower education, due to their own knowledge limitations, may lack healthy lifestyle values. They don't have strong motivation to establish and maintain a healthy lifestyle. Meanwhile, long working hours squeeze their time and opportunities for physical exercise and community participation, making them difficult to develop physical exercise habits and expand formal social interaction. Lack of channels to release stress causes a significant negative impact on their health too.

For those with a higher education level, especially those with a college degree or above, they are more likely to enter the primary labor market, engaging in more free and creative work and having relatively fewer adverse factors for health in the working environment. Also, their income returns are relatively high, which is conducive to creating healthy living conditions and lifestyles (increasing physical exercise). They have relatively stable work and have been easy to bring satisfaction and security to themselves. The reciprocal communication brought by physical exercise and group activity participation helps to release negative emotions in life and work.

Due to the limitation of data, we only use the frequency of physical exercise and group activity participation as indicators to measure people's lifestyles and social interactions which is not enough. Further research is needed to examine other lifestyles (such as smoking, drinking, vacation, physical examination, and diet). In addition, whether the social interaction network scale, structure, and other indicators can become the intermediary mechanism of education affecting health remains to be further analyzed and tested in future research.

## Figures and Tables

**Table 1:** Descriptive statistical results.

Variables	Mean Value	Standard Deviation	Min	Max
Self-rated health	0.769	0.422	0	1
Mental health	90.6	12.5	96	39
Level of education	2.957	1.255	1	5
Years of completed education	8.701	4.825	0	19
Gender	0.490	0.500	0	1
Registration place	0.302	0.459	0	1
Age	50.527	16.739	18	103
Personal annual income	8.029	3.884	0	16.111
Physical exercise	3.685	1.553	1	5
Group activities	4.447	1.104	1	5

**Table 2:** The mechanisms for the relationship between education and physical health.

Variables	Model 1	Model 2	Model 3	Model 4	Model 5
Years of completed education		0.127^*∗∗∗*^	0.102^*∗∗∗*^	0.103^*∗∗∗*^	0.105^*∗∗∗*^
		(3.83)	(3.48)	(3.65)	(3.23)
Gender	0.128^*∗∗∗*^	0.111^*∗∗∗*^	0.110^*∗∗∗*^	0.129^*∗∗∗*^	0.132^*∗∗∗*^
	(3.82)	(3.74)	(3.64)	(3.01)	(3.19)
Registration place	0.263^*∗∗∗*^	0.224^*∗∗∗*^	0.248^*∗∗*^	0.246^*∗∗*^	0.250^*∗∗∗*^
	(5.35)	(3.28)	(4.57)	(4.47)	(4.71)
Age	−0.063^*∗∗∗*^	−0.066^*∗∗∗*^	−0.059^*∗∗∗*^	−0.061^*∗∗∗*^	−0.062^*∗∗∗*^
	(−11.22)	(−11.77)	(−11.68)	(−11.65)	(−11.17)
Primary school	0.033				
	(1.34)				
Junior high school	0.122^*∗∗∗*^				
	(4.73)				
High school	0.153^*∗∗∗*^				
	(5.08)				
College and above	0.161^*∗∗∗*^				
	(4.69)				
Personal annual income		0.142^*∗∗∗*^	0.166^*∗∗∗*^		
		(5.85)	(4.58)		
Physical exercise		0.127^*∗∗∗*^		0.152^*∗∗∗*^	
		(5.34)		(4.22)	
Group activities		0.123^*∗∗∗*^			0.180^*∗∗∗*^
		(3.25)			(4.77)
Education × personal income			0.101^*∗∗∗*^		
			(3.80)		
Education × physical exercise				0.107^*∗∗∗*^	
				(3.73)	
Education × group activities					0.114^*∗∗∗*^
					(3.02)
Constant term	0.934^*∗∗∗*^	1.100^*∗∗∗*^	0.848^*∗∗∗*^	1.141^*∗∗∗*^	1.250^*∗∗∗*^
	(24.84)	(21.66)	(18.93)	(21.56)	(17.59)
Sample size	11,078	11,078	11,078	11,078	11,078
*R* ^2^	0.119	0.143	0.128	0.129	0.126

^1^The reference group comprises females, rural people, and people without any education. ^2^^*∗∗∗*^*p* < 0.01, ^*∗∗*^*p* < 0.05, ^*∗*^*p* < 0.1.

**Table 3:** The mechanisms for the relationship between education and mental health.

Variables	Model 1	Model 2	Model 3
Years of completed education		0.010^*∗∗∗*^	0.014^*∗∗*^
		(4.20)	(2.12)
Gender	0.001	0.014	0.015
	(0.07)	(1.14)	(1.16)
Age	−0.005^*∗∗∗*^	−0.005^*∗∗∗*^	−0.005^*∗∗∗*^
	(−10.30)	(−11.43)	(−10.95)
Registration place	0.060^*∗∗∗*^	0.022	0.017
	(4.03)	(1.47)	(1.12)
Primary school	0.025^*∗∗∗*^		
	(1.17)		
Junior high school	0.144^*∗∗∗*^		
	(5.01)		
High school	0.168^*∗∗∗*^		
	(5.19)		
College and above	0.179^*∗∗∗*^		
	(5.22)		
Personal annual income		0.019^*∗∗∗*^	0.034^*∗∗∗*^
		(6.56)	(5.39)
Physical exercise		0.027^*∗∗∗*^	0.058^*∗∗∗*^
		(6.62)	(4.56)
Group activities		0.014^*∗∗∗*^	0.029^*∗∗∗*^
		(6.33)	(5.02)
Education × personal income			0.002^*∗∗∗*^
			(3.28)
Education × physical exercise			0.003^*∗∗∗*^
			(2.58)
Education × group activities			0.001^*∗∗∗*^
			(3.17)
Constant term	0.987^*∗∗∗*^	1.078^*∗∗∗*^	1.039^*∗∗∗*^
	(25.70)	(24.68)	(13.45)
Sample size	11,078	11,078	11,078
*R* ^2^	0.126	0.151	0.156

^1^The reference group comprises females, rural people, and people without any education.^2^^*∗∗∗*^*p* < 0.01, ^*∗∗*^*p* < 0.05, ^*∗*^*p* < 0.1.

## Data Availability

Data available in Chinese General Social Survey, CGSS http://cgss.ruc.edu.cn/English/Home.htm.
